This article has been retracted.

# Image Effect Observation of Acanthopanax senticosus on Antifatigue Activity after Exercise

**DOI:** 10.1155/2022/7588680

**Published:** 2022-08-27

**Authors:** Xiangdong Zhang, Wanning Zhu

**Affiliations:** ^1^Beijing Normal University at Zhuhai, Zhuhai, Guangdong 519087, China; ^2^Sports Institute of Chengdu University of Technology, Chengdu, Sichuan 610059, China

## Abstract

In order to explore the effect of Acanthopanax senticosus on antifatigue activity after exercise, this paper proposes an image effect observation based on the effect of Acanthopanax senticosus on antifatigue activity after exercise. This method recommends key technical problems and solutions based on the information represented by image effect observation and explores the influence of Acanthopanax senticosus on antifatigue after exercise. Through the retrospective analysis of certain personnel, it is shown that the image effect observation based on the influence of Acanthopanax senticosus on the antifatigue activity after exercise is about 25% more accurate than the traditional method. Most of the active ingredients of Acanthopanax senticosus have phenolic hydroxyl groups, which can resist oxidation, fatigue, focus attention, and reduce work mistakes. This experiment shows that after sleep deprivation, the antioxidant capacity of the body decreases with time. Acanthopanax senticosus extract can significantly improve the above symptoms and fight fatigue.

## 1. Introduction

Fatigue is a comprehensive response to many physiological and biochemical changes in the body caused by multiple factors [1]. In 1982, the Fifth International Conference on exercise biochemistry defined it as follows: the physiological process of the body cannot maintain its function at a specific level or each organ cannot maintain its predetermined exercise intensity [2]. Fatigue is divided into physical fatigue and psychological fatigue. Physical fatigue is mainly manifested in the decline of sports ability, and psychological fatigue is mainly manifested in the negative changes of behavior and will. The process and mechanism of fatigue are very complex, and there are many theories to explain the mechanism of fatigue, such as the theory of energy exhaustion, the theory of metabolite accumulation, the theory of free radical increase, the theory of internal environment disorder, the theory of nerve fatigue, and the theory of body mutation [3]. These theories provide a theoretical basis for the prevention and treatment of fatigue and the study of its mechanism. However, due to the complexity of the fatigue process, various theories cannot fully explain the exact mechanism of fatigue, and different drugs have different mechanisms of alleviating fatigue, so in-depth research is needed.

With the increasing pressure of life, it has become a common phenomenon in contemporary society. Long-term sleep deprivation will have a significant impact on the central nervous system, accelerate the oxidative aging of the body, and aggravate fatigue. Sleep deprivation (SD) refers to a series of clinical symptoms caused by sleep loss in various pathological or physiological states [4]. With the gradual deepening of the global research on sleep deprivation, the phenomenon of sleep deprivation has gradually attracted attention, but at present, there are few reports on the effect of Acanthopanax senticosus on sleep-deprived human body.

Fatigue is a normal physiological phenomenon in a certain range [5]. With the development of society, the use of high technology has greatly improved the efficiency of work and life, and then, the pace of life has become faster and faster. The pressure from work, family, housing, medical treatment, interpersonal relations, and so on makes people in a state of tension for a long time, which is easy to cause physical fatigue and psychological fatigue. If it cannot be alleviated for a long time, it will turn into pathological fatigue, which will endanger people's physical and mental health and seriously degrade the quality of life. Therefore, looking for effective and safe antifatigue drugs has become a research focus of modern medicine. At the same time, the research on the mechanism of fatigue and the search for effective antifatigue drugs have also attracted extensive attention in sports medicine and military medicine. In the field of sports, athletes need to carry out long-term high-intensity training of physical strength, endurance, and strength in order to improve their performance in competitive sports. During the training process, a large amount of energy and materials are consumed, muscles continue to contract, and metabolites are accumulated, making the body in a state of fatigue, so it is difficult to achieve ideal sports performance. In the military field, military operations often need to be carried out in special environments, such as natural environments such as plateau hypoxic areas, cold areas, and hot areas, and special environments such as closed cabins and underground shelter projects. Most of the environment is bad, and affected by many composite factors such as high temperature, high humidity, noise, vibration, ionizing radiation, and harmful gases, the physical consumption and mental burden of officers and soldiers are increased. Long-term exposure to this environment will do harm to the physical and mental health of operators and may show fatigue symptoms such as inattention, anxiety, fatigue, endocrine disorders, and decreased immunity. This state will seriously affects the operational efficiency and combat effectiveness of military personnel. Therefore, the research of antifatigue drugs is also of great significance to military medicine [6].

At present, most of the antifatigue drugs on the market are chemical drugs, which not only play a good therapeutic effect but also bring great side effects. Traditional Chinese medicine has the characteristics of many active ingredients, mild effects, and small side effects. As an antifatigue drug, the research and development of traditional Chinese medicine has broad prospects [7]. Acanthopanax senticosus is the dry root and rhizome or stem of Acanthopanax senticosus, a plant belonging to Acanthopanax senticosus family. Its main pharmacodynamic components are saponins, lignans, and Echinacea polyphenols (eugenin and Acanthopanax senticosus glycoside E). Pharmacological experiments have verified that Acanthopanax senticosus has the effects of compression resistance, antiulcer, antitumor, anti-inflammatory, antiradiation, and liver protection.

Human internal psychological processes cannot be directly observed, and researchers can only infer the process in the brain based on the observed stimulus response. The research on the process of memory in the brain can only measure the coding form, storage capacity, retention time, and the conditions they depend on by measuring their performance or reaction time at a certain interval after human learning or performing a task. The foundation of learning and memory experimental methodology is conditioned reflex, from which various methods are derived, as shown in Figure 1.

## 2. Literature Review

Kkj et al. said that somatic fatigue can be divided into two types: peripheral fatigue and central fatigue [8]. Peripheral fatigue mainly refers to the fatigue of sports organ muscles, which is reflected in the decline of energy and material output power and muscle strength, that is, the decline of sports endurance. Bokp et al. said that exercise endurance is the most direct, objective, and powerful index to evaluate body fatigue [9]. Human models used to measure exercise endurance include treadmill model, swimming model, and pole climbing model. The running platform model equipment is expensive, which has great mechanical damage to human feet, and few people can measure it at the same time, which is not convenient for popularization. The climbing pole model device is simple, but some often jump down because they are unwilling to climb the pole, and uncontrollable factors such as the smoothness and scratch degree of the climbing pole will also affect the experimental results. Therefore, at present, swimming experiment with simple experimental device, no mechanical injury, mandatory, and good reliability of experimental results is the most extensive choice for sports endurance experiment.

Boehncke et al. showed through the experimental results that people have poor memory in the spatial resolution learning task of the rotating platform and found that their LTP effect is poor [10]. At the same time, they found that even among the same group, there was a significant correlation between people's memory ability and their LTP response intensity. Phillips et al. reported that the training process of conditioned reflex was accompanied by the change of LTP. They carried out ¥ maze learning training on people and found that the amplitude of group spike evoked by perforin fibers 4 hours and 24 hours after training was significantly higher than that before training. Among them, the LTP effect of people with good memory increased significantly, while the LTP effect of people with poor memory did not increase significantly [11]. Conversely, studies have shown that factors or drugs that affect LTP can also affect learning and memory processes. In conclusion, these data suggest that LTP may be the neural basis of learning and memory.

O'Neill et al. found that NE concentration increased and metabolism accelerated during REM sleep deprivation, and its transporter NE transporter located on the postsynaptic membrane also appeared in large numbers. It has the function of reingesting NE to maintain the relative reserves of NE in synapses and improve the efficiency of synaptic transmission [12]. The results showed that the concentration of NE in human hippocampus increased significantly after 48 hours of sleep deprivation and decreased significantly when sleep deprivation reached more than 96 hours, accompanied by a significant reduction in human learning ability.

There is excessive production of oxygen free radicals in brain tissue. Free radicals can cause degenerative changes in tissues and cells of the body and can cause abnormal lipid metabolism and produce excessive lipofuscin and MDA, thereby damaging the functions of cell membranes, organelles, and enzymes. SOD is a specific enzyme for the body to eliminate oxygen free radicals. The level of SOD can reflect the level of oxygen free radicals. The increase of SOD activity in brain tissue after sleep deprivation suggests that the content of oxygen free radicals in brain increases. Therefore, it is speculated that the increase of oxygen free radicals and the decrease of their scavenging ability may be one of the important reasons for the impairment of brain function and the decline of learning and memory ability after sleep deprivation.

Lee et al. believe that dopamine in the brain is related to maintaining muscle movement balance, affecting the secretion of some hormones in the pituitary gland and participating in mental activities. Brain dopamine plays an important role in controlling the process of exercise. With the emergence of exercise-induced fatigue, the content of pivot tends to decrease [13]. The concentration and activity of dopamine in the brain decrease, which reduces the coordination ability of muscle activities, leading to fatigue. Zhao et al. found in the experiment that the increase of brain 5-htida ratio can lead to exercise-induced fatigue by weakening the level of promotion and the loss of motor nerve coordination [14].

## 3. Method

### 3.1. Evaluation Index

In order to fairly compare different algorithms in the field of image segmentation, there must be standard and widely recognized indicators for evaluation. The commonly used evaluation criteria for medical image segmentation algorithms are accuracy, recall, specificity, Dice coefficient, and Jaccard index. *A* is the true annotation of a medical image, and *B* is the prediction result of the segmentation model. Then, the accuracy AC, recall SE, specificity SP, Dice coefficient DSC, and Jaccard index JAC are expressed, respectively, as shown in the following formulas:

(1) $$\begin{array}{c} \text{AC}=\frac{\text{TP}+\text{TN}}{\text{TP}+\text{TN}+\text{FP}+\text{FN}}, \end{array}$$

(2) $$\begin{array}{c} \text{SE}=\frac{\text{TP}}{\text{TP}+\text{FN}}, \end{array}$$

(3) $$\begin{array}{c} \text{SP}=\frac{\text{TN}}{\text{TN}+\text{FP}}, \end{array}$$

(4) $$\begin{array}{c} \text{DSC}=\frac{2\left(A\cap B\right)}{A+B}, \end{array}$$

(5) $$\begin{array}{c} \text{JAC}=\frac{A\cap B}{A\cup B}, \end{array}$$

Accuracy refers to the percentage of correctly predicted pixels in the total pixels. In the case of unbalanced categories, it cannot be used as a good indicator to measure the segmentation results [15, 16]. Recall rate, also known as sensitivity, only focuses on the proportion of true labels correctly predicted, while the focus on specificity is just the opposite. These two indicators are relatively sensitive to the size of segmentation targets [17]. Dice coefficient is the most commonly used evaluation index in the task of medical image segmentation, which can better avoid the problem of category imbalance in the field of medical image. Jaccard index is also called intersection union ratio (IoU), and its relationship with Dice coefficient is shown in the following formula:

(6) $$\begin{array}{c} \text{DSC}=\frac{2\text{JAC}}{1+\text{JAC}}. \end{array}$$

In practical applications, we often choose the above evaluation indicators according to the needs and prove the accuracy and stability of the segmentation algorithm from multiple dimensions.

### 3.2. Uniform Design

The commonly used uniform design table is that *n* is an odd number table. According to the literature, when *n* is an even number, the uniform design table is an odd number uniform design table with *n* + 1 removed from the last row [18]. Therefore, the experimental design table of 3 factors and 8 levels is obtained by crossing out the last row on the basis of the uniform design table and selecting columns 1, 3, and 5 at the same time, as shown in Tables 1 and 2.

According to the experimental arrangement in Tables 1 and 2, weigh different amounts of Acanthopanax senticosus, Astragalus membranaceus, and Codonopsis pilosula, and get 8 compounds with different proportions. Eight different compounds were soaked in 8 times the amount of water for 0.5 h and extracted three times with a condensing reflux device for 2 h each time. The extracts were combined, reduced with pressure, and concentrated with a rotary evaporator, and the concentrated solution was dried to obtain the extract [13, 19].

The results of uniform design experiment were statistically processed by uniform design u 3.00 software, and regression analysis was carried out by full regression method. The significance level was *α* = 0.05. The results of human weight-bearing swimming experiment were statistically processed by the SPSS 18.0 software. All data were expressed in XTS. The time of exhausted swimming was analyzed by one-way ANOVA. The differences between groups were compared by LSD-t method, and the significance level was *α* = 0.05.

In the retrospective analysis, the personnel in each group were in good condition without any adverse reactions. There was no significant difference between the body weight at the beginning of the analysis and the body weight at the end of the experiment, as well as the weight increased during the experiment, indicating that the compound with different proportions had no significant effect on the growth of body weight.

The compatibility of Acanthopanax senticosus, Astragalus membranaceus, and Codonopsis pilosula has a good antifatigue effect by harmonizing the five internal organs and warming and cooling. In this section of the experiment, the uniform design method was used to arrange the experiment, and the best dose ratio relationship of the compound was investigated with the exhaustion swimming time in the endurance experiment as the evaluation index. Through visual analysis of the experimental results, it was found that the exhaustion swimming time of the two groups with the ratio of 30 : 21 : 7 and 3 : 1 : 1 was the longest [20, 21]. From the regression equation *Y* = 8.46 + 0.184*X*; +0.739*Xz* − 0.194*X*, it can be seen that the coefficients of *X* and *X* are positive, indicating that the exhausted swimming time increases with the increase of the dosage ratio of Acanthopanax senticosus and astragalus, while the coefficient of *X*3 is negative, indicating that the exhausted swimming time decreases with the increase of the dosage ratio of Radix Codonopsis. The absolute value of partial regression coefficient *x*2 > *x*3 > *x*1 shows that the primary and secondary order of the influence of the three drugs on swimming time is Astragalus membranaceus>Acanthopanax senticosus>Codonopsis pilosula. Therefore, when determining the optimal experimental scheme, within the specified dose range, the dosage ratio of Acanthopanax senticosus and Astragalus should be higher than the upper limit, and the dosage ratio of Codonopsis pilosula should be lower than the lower limit, that is, Acanthopanax senticosus 30 g, Astragalus 30 g, and Codonopsis pilosula 6 g, which is basically consistent with the trend of intuitive analysis. At the same time, the optimization results of uniform design also showed that when Acanthopanax senticosus 30 g, Astragalus 30 g, and mingdangshen 6G, that is, when the ratio is 5 : 5 : 1, the effect of delaying fatigue is the best. The original formula of the compound 3 : 2 : 1 also has a better effect of alleviating fatigue. Whether the optimized formula has a better effect of alleviating fatigue than the original formula needs to be verified in the next step.

At present, Morris water maze has been widely used in the study of neurobiological mechanism of learning and memory and neuropharmacology because of its reasonable design. It is mainly used to study the measurement of spatial learning and memory ability and working memory of experimental human body. The classic water maze experiment includes location navigation experiment and spatial search experiment. The former measures adult learning ability, and the latter measures adult memory ability. Compared with platform jumping, avoiding darkness, and other detection tools, its main advantages include the following: it can provide more experimental parameters, systematically and comprehensively investigate the process of spatial cognitive processing of experimental human body, and objectively reflect its cognitive level. The learning and memory disorders of the experimental human body are separated from sensory and motor defects, so as to reduce their interference to the detection of learning and memory process; the operation is simple, and the data error is small. It has reliable sensitivity to age-related spatial memory impairment and is a particularly useful tool for judging people's spatial learning ability. The disadvantage is that there are many factors to be considered in the design of the experimental procedure, which requires the experimenter to have a certain knowledge of neurobiology, cognitive psychology, and mathematical statistics. Its statistical analysis is more complex: it is insensitive to the slight decline of learning and memory ability; immersing the human body in water may cause endocrine or other stress reactions. Due to too much physical exertion, it is difficult for people who lose too much body temperature to complete the task; there are high requirements for experimental conditions, so it is necessary to keep the spatial clues provided by the objects around the maze fixed, the water temperature should be kept constant, and it is also important to keep quiet and consistent light during the experiment [22, 23].

The hexagonal maze box experimental device has been proved to be an effective learning and memory test tool through a large number of experiments. The maze combines the advantages of the above experimental methods: for example, it can quantify human behavior, provide more experimental parameters, and systematically and comprehensively investigate human cognitive process. Objectively reflect the cognitive level of the human body. Active avoidance and passive avoidance can be observed at the same time. It can detect both spatial reference memory and spatial working memory. It can record the search route of human body and reflect its search strategy. It will not consume too much physical strength.

The above behavioral methods can evaluate the learning and memory of the subjects as a whole. With the continuous deepening of the study of learning and memory and the emergence of various new theories of learning and memory, new experimental models and advanced experimental technology are applied to the research, which also poses new challenges to the study of learning and memory. Therefore, how to combine the traditional behavioral methods with the latest technical means to provide more scientific, accurate, and intuitive data for the study of learning and memory has become a problem that must be solved in the field of behavioral research in the future. The results of human hexagonal maze are shown in Figure 2.

The results showed that compared with the large platform control group, the search frequency of each group after sleep deprivation was significantly increased, and the search time was shortened. Among them, each dose group of Acanthopanax senticosus was shorter than that of the sleep deprivation group. Compared with the large platform control group, the number of errors in the sleep deprivation group was significantly increased and the cognitive rate was reduced (*p* < 0.01). Compared with the sleep deprivation group, the cognitive rate was increased in each dose group of Acanthopanax senticosus, and the difference between the high- and medium-dose groups was extremely significant (*p* < 0.01), and the difference between the low-dose group was significant (*p* < 0.05).

Neurophysiological methods can record electrophysiological signals of the central nervous system at different levels by using a variety of techniques, such as detection of electrical signals of the nervous system, induction of electrical signals of synaptic circuits of neurons, microelectrode recording, and patch clamp, for example, the electrical signals of cerebral cortex, the potential signals of neuronal groups in various brain tissues, the membrane potential signals of single nerve cells, and the current signals of ion channels on the membrane of nerve cells. Analyze the changes of these electrophysiological signals under the action of drugs, so as to study the effect and mechanism of drugs [24].

Neurophysiological research (from whole to ion channel) has multiple levels of methods, but it can be roughly divided into two categories: in vitro and in vivo. Among them, brain tissue slice in vitro incubation method and patch clamp ion channel method belong to in vitro research methods. The advantages of these methods are as follows: there is no blood-brain barrier, the components of perfusate can be changed flexibly, the speed of drug application and elution is fast, it is easy to control the concentration of perfusate drugs to establish a dose-response relationship, and it can clearly observe the morphology of nerve tissue or nerve cells, and correctly grasp the drug action site and signal detection site. We can observe the response of the single synaptic circuit cell population of the nervous system to the single ion channel of the nerve cell membrane at different levels. However, in vitro research methods, cut off the normal synaptic connection between brain slices and surrounding tissues and affect various regulatory factors, which may change some response characteristics of neurons. Moreover, in vitro research methods require the use of relatively single drug components, which is especially suitable for the study of the action mechanism of agonists and antagonists of various nerve receptors. For the crude extract or Decoction of traditional Chinese medicine, it will interfere with the evaluation of in vitro experimental results due to the influence of impurities and physical and chemical properties (impurity particles, pH of drugs, etc.).

## 4. Results and Analysis

A certain number of personnel were selected for retrospective analysis. During the analysis, all groups were in good condition without any adverse reactions. The weight changes of people in different groups are shown in Table 3. It can be seen from the table that there is no significant difference between the weight of people at the beginning of the experiment and the weight at the end of the experiment, as well as the weight increased during the experiment, indicating that different drugs have no significant impact on the growth of human weight [25].

According to the results of human weight-bearing swimming experiment in Table 4, compared with the blank group, the positive drug group, the ratio of 3 : 2 : 1 group, and the ratio of 5 : 5 : 1 group all prolonged the exhaustion swimming time of people to varying degrees, with significant difference (*p* < 0.05), as shown in Table 4.

Exhaustive swimming time is the simplest and most intuitive index in sports endurance experiment. In the validation experiment, the compound extract with the ratio of 3 : 2 : 1 and the compound extract with the ratio of 5 : 5 : 1 showed better antifatigue effect, and there was a significant difference between the two groups. However, there is no significant difference in the effect of alleviating fatigue between the two proportions. Because the original prescription ratio of 3 : 2 : 1 is the clinical experience prescription of the hospital, its effectiveness and safety are good, and the proportion of Astragalus in this ratio is small, and the cost is relatively low.

Fatigue is the result of multiple factors. The most direct and objective performance is the reduction of muscle contractility, the decline of exercise endurance, and the emergence of exhaustion. The length of exhaustive swimming is the most direct behavioral indicator of exercise endurance in human weight-bearing swimming experiments. The analysis of exhaustion swimming time shows that the total extract HD group, 40% ethanol and 75% ethanol elution site HD group, has a longer exhaustion swimming time, which has a significant difference compared with the blank group. Among them, the total extract HD group has the best effect, indicating that the compound total extract has a better antifatigue effect.

The process of fatigue is complex, and the specific mechanism is not clear. At present, the more recognized mechanisms are energy exhaustion theory, metabolite accumulation theory, internal environment disorder theory P, etc. According to the above different theories, four representative biochemical indicators, TG, bun, LDH, and CK, are selected for detection. If two or more indicators are positive, it indicates that the tested drug has antifatigue effect.

## 5. Conclusion

Due to the influence of various social factors such as high work pressure, fast pace of life, high consumption level, and special working environment such as high temperature, high humidity, noise, harmful gases, and ionizing radiation, fatigue in various fields is becoming more and more serious, and more and more people are tired. Therefore, fatigue has become the research focus of social medicine, sports medicine, military medicine, preventive medicine, and other disciplines. Acanthopanax senticosus replenishes Qi, invigorates the spleen, invigorates the kidney, and calms the nerves. Astragalus membranaceus can not only tonify the spleen but also elevate the middle Qi, brighten Codonopsis pilosula, nourish yin and stomach, and calm the liver and detoxify. The three prescriptions are warm and cool, regulate and tonify the liver and kidney, and take into account the spleen and stomach, which is consistent with the understanding of traditional Chinese medicine on the pathogenesis of fatigue, and this prescription has been used in hospitals as a hospital preparation to treat fatigue. Therefore, this study is guided by pharmacological activity to find an effective part against fatigue caused by continuous exercise, further study the effect of this part on fatigue in special environment, and preliminarily analyze its antifatigue material basis.

In the experiment of optimizing the proportion of compound Acanthopanax senticosus, the compounds with different proportions were obtained through uniform design. Through the human weight-bearing swimming experiment, the optimal proportion of antifatigue effect was found with the exhaustion swimming time as the evaluation index. The results showed that the extracts with the ratio of 30 : 21 : 7 and 3 : 1 : 1 significantly prolonged the exhaustion time. The regression equation *Y* = 8.46 + 0.184*X*_1_ + 0.739*X*_2_ − 0.194*X*_3_ was obtained by using the uniform design software. The equation was significant. On this basis, the optimal ratio was optimized to be 5 : 5 : 1. The original formula of compound Acanthopanax senticosus is 3 : 2 : 1. Comparing it with the effect of the extract with the optimal ratio on people's swimming time, it is found that there is no significant difference in the antifatigue effect of the two formulas. As an empirical formula, the original formula of 3 : 2 : 1 has better effectiveness and safety, and the cost is relatively low, so it is the optimal compatibility ratio after comprehensive consideration. The best proportion of antifatigue effect of compound Acanthopanax senticosus was confirmed, the best extraction method was determined, and the effective parts for resisting fatigue caused by continuous exercise and alleviating fatigue in special environment were screened through in vivo experiments. The main pharmacodynamic components of the effective parts were determined based on liquid chromatography-mass spectrometry, and the safety of the effective parts was evaluated, and no obvious acute toxicity was found.

## Figures and Tables

**Figure 1:** Basic principle of research method for memory process in brain.

**Figure 2:** Human hexagonal maze performance.

**Table 1:** Level of uniform design factors.

Level/factor	1	2	3	4	5	6	7	8
(A) Acanthopanax senticosus (g)	9	12	15	18	21	24	27	30
(B) Astragalus (g)	9	12	15	18	21	24	27	30
(C) Dangshen (g)	6	7	8	9	10	11	12	13

**Table 2:** Three-factor eight-level uniform design.

Experiment No.	Acanthopanax senticosus	Astragalus membranaceus	Dangshen of Ming Dynasty
1	1 (9)	4 (18)	7 (12)
2	2 (12)	8 (30)	5 (10)
3	3 (15)	3 (15)	3 (8)
4	4 (18)	7 (27)	1 (6)
5	5 (21)	2 (12)	8 (13)
6	6 (24)	6 (24)	6 (11)
7	7 (27)	1 (9)	4 (9)
8	8 (30)	5 (21)	2 (7)

**Table 3:** Effects of different proportions of compound Acanthopanax senticosus on human body weight (*n* = 10).

Group	Initial weight (g)	Final weight (g)	Increased weight (g)
Control	22.37 ± 1.20	31.19 ± 1.28	8.82 ± 0.57
Red ginseng	22.22 ± 0.96	31.21 ± 1.06	8.99 ± 0.60
3 : 2 : 1	22.19 ± 1.08	31.86 ± 1.52	9.67 ± 0.77
5 : 5 : 1	22.41 ± 0.71	31.41 ± 1.85	9.00 ± 1.21

**Table 4:** Effects of different proportions of compound Acanthopanax senticosus on human exhaustion swimming time (*n* = 10).

Group	Dose (mg/kg)	Swimming time (min)
Control	-	9.17 ± 2.45
Red ginseng	200	12.95 ± 4.21^∗^
3 : 2 : 1	500	14.03 ± 5.25^∗^
5 : 5 : 1	500	14.75 ± 5.43^∗^

## Data Availability

The data used to support the findings of this study are available from the corresponding author upon request.

## References

[1] Choi R. J., Jlcr B., Sfr C. (2021). Usability testing of tablet-based cognitive behavioral intervention application to improve a simple walking activity for older adults with arthritis fatigue. *Geriatric Nursing*.

[2] Sander C., Braun N., Modes F., Schlake H. P., Hildebrandt H. (2022). Can biofeedback-based training alleviate fatigue and vigilance performance in fatigued MS patients. *Neuropsychological Rehabilitation*.

[3] Monteiro T. G., Skourup C., Zhang H. (2021). A task agnostic mental fatigue assessment approach based on EEG frequency bands for demanding maritime operation. *IEEE Instrumentation and Measurement Magazine*.

[4] Goedendorp M. M. (2022). It is improbable that high intensity exercise reduces fatigue during chemotherapy. *BMJ*.

[5] Leaviss J., Davis S., Ren S., Hamilton J., White P. (2020). Behavioural modification interventions for medically unexplained symptoms in primary care: systematic reviews and economic evaluation. *Health Technology Assessment*.

[6] Ali A. M., Kunugi H. (2021). Screening for sarcopenia (physical frailty) in the COVID-19 era. *International Journal of Endocrinology*.

[7] Turri-Silva N., Ricci-Vitor A. L., Cipriano G. (2020). Functional resistance training superiority over conventional training in metabolic syndrome: A randomized clinical trial. *Research Quarterly for Exercise and Sport*.

[8] Jensen K. K., Brøndum T. L., Leerhøy B. (2020). Preoperative, single, high-dose glucocorticoid administration in abdominal wall reconstruction: a randomized, double-blinded clinical trial. *Surgery*.

[9] Kahraman B. O., Savci S., Ozsoy I. (2020). Effects of neuromuscular electrical stimulation in patients with pulmonary arterial hypertension: a randomized controlled pilot study. *Journal of Cardiology*.

[10] Ritchlin C. T., Mease P. J., Boehncke W. H. (2022). Sustained and improved guselkumab response in patients with active psoriatic arthritis regardless of baseline demographic and disease characteristics: pooled results through week 52 of two phase iii, randomised, placebo-controlled studies. *RMD Open*.

[11] Phillips S. M., Welch W. A., Fanning J. (2020). Daily physical activity and symptom reporting in breast cancer patients undergoing chemotherapy: an intensive longitudinal examination. *Cancer Epidemiology Biomarkers & Prevention*.

[12] O'Neill C. T., Proietti T., Nuckols K., Clarke M. E., Walsh C. J. (2020). Inflatable soft wearable robot for reducing therapist fatigue during upper extremity rehabilitation in severe stroke. *IEEE Robotics and Automation Letters*.

[13] Lee M. C., Hsu Y. J., Ho C. S., Chang C. H., Chiang W. D. (2021). Evaluation of the efficacy of supplementation with planox lemon verbena extract in improving oxidative stress and muscle damage: a double-blind controlled trial. *International Journal of Medical Sciences*.

[14] Zhao Y., Li T. G., Pu R., Shui L., Chen Y. S. (2020). Effect of moxibustion on body weight and peripheral and cerebral cortical IL-6 and IL-10 levels in fatigue rats. *Zhen ci yan jiu= Acupuncture Research*.

[15] Li S., Pan H., Wang Y., Sun J. (2020). Polyelectrolyte complex-based self-healing, fatigue-resistant and anti-freezing hydrogels as highly sensitive ionic skins. *Journal of Materials Chemistry A*.

[16] Ding W., Li X., Yang H., An J., Zhang Z. (2020). Utilizing statistical information for interval analysis: a method for analyzing the interval uncertainty of line-of-sight measurement error of space-borne observation platforms. *IEEE Access*.

[17] Jia L., Zhao F. (2022). Evaluation of silymarin extract from Silybum marianum in mice: anti-fatigue activity. *Food Science and Human Wellness*.

[18] Nagy M., O'Sullivan M., Block S., Hasson R. E. (2020). Acute effects of intermittent physical activity on perceptions of exercise-related fatigue in children. *Journal of Physical Activity & Health*.

[19] Lin Y. K., Wu B. H., Lin Y. H., Chan S. T., Chiang C. F. (2022). Effects of supplementation with ginseng and branched chain amino acids improved central fatigue and enhanced attention during exercise: a randomized, double-blind, placebo controlled. *Journal of Food and Nutrition Research*.

[20] Hsu W. L., Chen C. P., Nikkhoo M. (2020). Fatigue changes neck muscle control and deteriorates postural stability during arm movement perturbations in patients with chronic neck pain. *The Spine Journal*.

[21] Fan M., Sharma A. (2021). Design and implementation of construction cost prediction model based on SVM and LSSVM in industries 4.0. *International Journal of Intelligent Computing and Cybernetics*.

[22] Rajendran A., Balakrishnan N., Ajay P. (2021). Deep embedded median clustering for routing misbehaviour and attacks detection in ad-hoc networks. *Ad Hoc Networks*.

[23] Li L., Diao Y., Liu X. (2014). Ce-Mn mixed oxides supported on glass-fiber for low-temperature selective catalytic reduction of NO with NH_3_. *Journal of Rare Earths*.

[24] Huang R., Zhang S., Zhang W., Yang X. (2021). Progress of zinc oxide-based nanocomposites in the textile industry. *IET Collaborative Intelligent Manufacturing*.

[25] Gu J., Wang W., Yin R., Truong C. V., Ganthia B. P. (2021). Complex circuit simulation and nonlinear characteristics analysis of GaN power switching device. *Nonlinear Engineering*.

